# Organoid Models for Salivary Gland Biology and Regenerative Medicine

**DOI:** 10.1155/2021/9922597

**Published:** 2021-08-27

**Authors:** Chen Zhao, Cuida Meng, Na Cui, Jichao Sha, Liwei Sun, Dongdong Zhu

**Affiliations:** Department of Otolaryngology Head and Neck Surgery, China-Japan Union Hospital of Jilin University, Changchun, China

## Abstract

The salivary gland is composed of an elegant epithelial network that secrets saliva and maintains oral homeostasis. While cell lines and animal models furthered our understanding of salivary gland biology, they cannot replicate key aspects of the human salivary gland tissue, particularly the complex architecture and microenvironmental features that dictate salivary gland function. Organoid cultures provide an alternative system to recapitulate salivary gland tissue in vitro, and salivary gland organoids have been generated from pluripotent stem cells and adult stem/progenitor cells. In this review, we describe salivary gland organoids, the advances and limitations, and the promising potential for regenerative medicine.

## 1. Introduction

Three major salivary glands (the parotid, submandibular, and sublingual glands) and numerous minor ones located in the upper aerodigestive tract produce saliva by a wide range of environmental and biological stimuli. Like most exocrine glands, salivary glands undergo their morphogenesis during the embryonic period when the branched ductal structures originate from an initial epithelial placode and grow into the mesenchyme [1]. The branched ductal structure comprises acinar, ductal, and myoepithelial cells. Acinar cells are responsible for protein and fluid secretion upon parasympathetic neuron stimulation, while ductal cells form a tubular conduit for saliva transportation and slight modification of ionic composition. Acini are wrapped by contractile myoepithelial cells inside the basement membrane embedded in the stroma containing immune cells, vasculature, and nerves [2]. The epithelial-mesenchymal crosstalk guides the morphogenesis of the salivary glands [3]. Any impairment to the architecture and/or function of the salivary glands may result in hyposalivation, manifested as xerostomia or “dry mouth syndrome” [4, 5]. The situation can be caused by systemic diseases including, but not limited to, Sjögren's syndrome, uncontrolled diabetes mellitus, and granulomatous diseases, however, more frequently by radiotherapy for head and neck cancer (HNC) [6, 7]. Patients with xerostomia suffer from swallowing and speaking difficulties, as well as oral and dental infections, each of them is life-disrupting. However, current therapeutic options mainly rely on artificial substitutes and systemic sialogogues, but they provide only temporary relief, not long-term benefits.

Three-dimensional architecture is the cornerstone of morphogenesis, and functional differentiation has been accepted during the last several decades, with the simultaneous advent of in vitro 3D culture technologies, and they enabled the generation of “organoids.” Organoids can be established from adult stem cells (ASCs) and pluripotent stem cells (PSCs), including induced pluripotent stem cells (iPSCs) and embryonic stem cells (ESCs) [8]. When placed into a hydrogel with an appropriate exogenous factor cocktail, stem cells develop into several cell types through cell sorting and lineage commitment that mimic the process in vivo. Since their remarkable ability reflects the properties of organs structurally and functionally, organoids are utilized to model organ development and diseases, drug discovery, and personalized therapy; meanwhile, they also shed light on regenerative medicine [9]. Increasing studies indicate that they are potential sources for regeneration of new salivary gland units. In this review, we will summarize the current literature concerning salivary gland organoid, the development of technology, the emerging roles in understanding salivary gland morphogenesis, and their great potential use in regenerative medicine. Furthermore, challenges to salivary gland organoid research and future directions are discussed.

## 2. Salivary Gland Development, Homeostasis, and Regeneration

To produce sufficient saliva within a limited space of the craniofacial complex, the salivary glands need to maximize the surface area to volume ratio during morphogenesis. This is realized by the programmed formation of interconnected and branched secretory acinus and ductal structures, which are highly similar in rodents and human. Most of our knowledge of salivary gland development come from ex vivo cultures of mouse embryonic submandibular glands [10, 11]. At mouse embryonic day (E) 11.5, the oral epithelium thickens and invaginates into the condensed mesenchyme, which is the beginning of salivary gland formation. Branching morphogenesis occurs during E12.5-14.5, and single epithelial bud sequentially undergoes several branching cycles, including bud enlargement, cleft formation, and terminal bud expansion. At E13, axons elongate along the epithelial cells and envelop the newly formed terminal buds, which finally differentiate into secretory acini. At E14.5, KRT19^+^ duct progenitor cells begin to proliferate and lead to duct extension; meanwhile, they condense at the midline and microlumen fuse to form a contiguous lumen [12]. Tubulogenesis ends at E18.5, and in parallel, proacinar cells mature with the hallmark of mucin protein production. This complex morphological transformation is rigorously regulated by multiple epithelial-mesenchymal crosstalks via growth factors (i.e., FGF, EGF, EDA, BMP, Wnt, and Hedgehog) and neurotransmitter- (i.e., acetylcholine and vasoactive intestinal peptide-) mediated signaling pathways [13]. However, the exact functions of each signaling molecule are difficult to define because epithelial arborization is an integrated process including cell duplication, branch point generation, and finally branch elongation.

Studies focusing on salivary gland cell proliferation and differentiation utilizing bromodeoxyuridine and ^3^H-thymidine labeling have accumulated evidences that stem cells play an important role in maintaining salivary gland homeostasis [14, 15]. These putative stem cells are mainly distributed to the excretory and intercalated ducts and maintain the morphological and molecular characteristics of undifferentiated stem cells [16]. Researchers have identified these putative stem/progenitor cells relied on the expression of c-Kit (CD117), keratin 5 (K5), keratin 14 (K14), Ascl3, CD24, CD29, and CD49f, based on molecular markers identified in other tissues and lineage tracing assays [17–21]. The label retaining cell (LRC) assay demonstrated that LRC, which are considered to be slow-cycling stem cells, colocalize with several stem cell markers, without obvious overlapping with each other, indicated that stem/progenitor cells of salivary glands are heterogeneous [22]. Their stemness of self-renewal and differentiation into acinar, ductal, and myoepithelial cells has been verified in vitro; however, the differentiation capacity in vivo needs to be further identified, especially in irradiated glands [17, 18, 21, 23]. Radiation hampers the replacement capacity of primitive stem cells by classical mitotic cell death, preventing their supplement to damaged secretory epithelia, a process generally irreversible [15]. However, after injuries such as main excretory duct ligation, the remaining intact duct is the source of stem cells leading to regeneration and substitution of excretory cells after ligation removed [24]. A recent fate-mapping experiment [25] revealed that differentiated acinar cells still self-duplicate, with relatively less contribution of stem/progenitor cells maintaining homeostasis [26]. The roles of distinct putative stem/progenitor cells as well as differentiated cells contribute to homeostasis remain to be clarified with the consideration of conditions.

## 3. Salivary Gland Organoids

### 3.1. Establishment of Salivary Gland Organoid Models

Salivary gland organoids are commonly established from fragments of mouse or human salivary glands dissociated utilizing mechanical and/or enzymatic digestion and then embedded in reconstructed ECM-like material, traditionally animal tissue derived protein extracts, such as Matrigel, fibrin gel, and collagen gel [27, 28] (Figure 1). Dispersed salivary gland cells develop and self-assembly into acini and/or ductal-like structures that express subsets of critical lineage markers. While organoids derived from rodent salivary gland are popular because our knowledge of salivary gland development mainly depends on rodent cells ex vivo cultures, human organoids derived from biopsies and resected salivary glands of preirridiation head and neck cancer surgical patients provide increasing information of human development biology. Importantly, distinct salivary gland stem/progenitor cells demonstrate different organoid formation abilities [17, 21, 29, 30]. Abundant studies provide proof of concept that fully functional regeneration of the salivary glands that can be achieved by reciprocal epithelial and mesenchymal interactions reproducing mimicking that during embryogenesis [31–33]. However, relatively less information of specific niche factors that promote the differentiation and formation of salivary gland organoids from pluripotent stem cells is far from clear, and several groups have succeeded in taking the first step [28, 33].

#### 3.1.1. Salivary Gland Organoids Generated from Pluripotent Stem Cells

PSCs can undergo differentiation into various cell lineages when induced by signals positioning and patterning the way during embryogenesis. Organoids generated from PSCs were first developed for brain by Lancaster and Knoblich, after acquisition neuroectoderm from embryoid bodies (EBs) ,and they generated them into organoids in spinning bioreators [34]. The protocol is pattern growth factors independent and thus gives PSCs the most freedom to self-organize. Since then, organoids generated from the endoderm, mesoderm, and ectoderm-derived PSCs were reported, including intestine, stomach, liver, pancreas, lung, and kidneys [35–40]. Aiming to replicate salivary gland development in vitro, Ogawa team has succeeded in differentiating mouse embryonic salivary gland epithelial cells into functionally mature gland germs with embryonic mesenchymal cells [41]. The organ germ underwent sequential branching morphogenesis, stalk elongation, and cleft formation after 3 days culture. However, this early approach was performed in 2D culture without 3D information for salivary gland development in vitro. The first attempt to differentiate PSCs into 3D salivary gland tissue that recapitulated embryonic salivary gland features was the establishment of organ rudiment cultures by Tanaka and colleagues that introduced a step-wise method [28]. Sox9 and Foxc1 are identified as essential organ-inductive transcriptional factors inducing oral epithelium (OE) thickening during initial stage of salivary gland development. Thus, after mouse submandibular ESCs' derived EBs are inducted into OE with cytokines (i.e., BMP4, SB-431542, LDN-193189, and FGF2), the forced expression of Sox9 and Foxc1 induce primitive OE to develop into branching structures, namely, salivary gland rudiment, composed of AQP5^+^ acinar-like cells, CK18^+^ ductal-like cells, and *α*-SMA^+^ myoepithelial-like cells after 15 days culture (Figure 2). On orthotopical transplantation into parotid gland-defective mice, the rudiment developed into tissue exhibiting mature salivary gland features. While groundbreaking, ESCs' inaccessibility for the human tissues is a concern that cannot be ignored, hampering the translational application of the model.

#### 3.1.2. Salivary Gland Organoids Generated from Adult Stem/Progenitor Cells

Early studies by Aileen and colleagues, in which fragments of rat submandibular gland were cultured in three-dimensional collagen gel matrix, led to maintained topological organization of the parent tissue; however, the outgrowth of these cultures was accompanied by central necrosis which led to a short surviving period [42]. Self-renewing salivary gland organoids during long-term culture were reported by Lombaert and colleagues in 2008. When cultured in rat tail collagen, isolated cells from rodent submandibular glands formed salispheres expressing stem cell markers including c-Kit, Sca-1, and Musashi; moreover, these salispheres were able to proliferate and differentiate towards acinar and ductal cells both in vitro and in vivo [17]. Enrichment of c-Kit^+^ cells in primary and secondary salispheres suggests that this three-dimensional sphere is a feasible way to concentrate salivary gland adult stem cells. Feng [29] reported the striking similarities of primitive human salivary gland stem cells to form organoids that differentiate into acinar and ductal lineages in collagen type I. The expansion of adult salivary gland organoids was enabled by culture conditon optimization. In addition to the cytokines such as FGF, Wnt3a, and R-spondin 1, which had been described to be important for organogenesis, regeneration and development of salivary glands [43, 44] and Alk (also known as TGF-*β*/Smad) signaling inhibitors were supplemented in the culture condition to suppress squamoid differentiation. This protocol was adapted to generate organoids from healthy human salivary glands and to recapitulate inflammatory diseases such as sialadenitis [45].

It is well known that in contrast to pluripotent stem cells, adult stem cells are difficult to proliferate and expand. Since salivary gland stem cell organoids shed light on autologous transplantation to restore irradiated salivary gland function, getting potent enough and sufficient stem cells for organoid establishment is the first problem to be addressed. Nanduri [46] reported an enhanced regenerative potential of cells derived from murine salispheres by selection of CD24^hi^CD29^hi^ subset, and an exciting 4-fold increased number of selected cells was generated after seven passages compared to expansion from unselected population. Similarly, using multiple surface markers, Xiao [47] identified Lin^−^CD24^+^c-Kit^+^Sca1^+^ a highly enriched population of adult salivary gland stem cells, and in vivo serial transplantation studies demonstrated self-renewal and multipotency of their progenies for at least 6 months after initial isolation.

### 3.2. Salivary Gland Organoids for Development and Morphogenesis

Branching morphogenesis is the key developmental process for salivary glands and other glandular organs including kidney, mammary gland, and lungs [48]. One hallmark of organoid models that the composition completely separated from the adjacent ECM ensures their efficiency of attempting to study the physical and chemical properties' roles of ECM in morphogenesis. In fact, organoids have been successfully used to study salivary gland epithelial branching morphogenesis. Using embryonic submandibular gland single epithelial cells cocultured in Matrigel with bone marrow-derived mesenchymal cells (MSCs), Farahat [32] demonstrated that MSCs induced a self-assembly organoid with branching morphology, and the process was sensitive to the initial cell ratio and total number, but growth factors are independent. Another study identified laminin-111 and FGF2, but not EGF, as niche factors that driven epithelial progenitor cell development into terminal buds displaying the robust AQP5 expression [27]. Organoids have also been applied to investigate salivary stem/progenitor cells as a branching driver. For instance, Coppes and colleagues have expanded single adult stem cells into an organoid with distinct lobular or ductal/lobular structures in a short-term culture manner [46]. In their follow-up study, robust Wnt signaling activation by the addition of R-spondin and Wnt3A guaranteed a long-term expansion of organoids comprising all the differentiated cell types [49]. These various organoid models investigated both human and rodent salivary gland branching morphogenesis, although recapitulated some, but not all aspects of that observed in vivo.

To realize the primary function of the salivary gland to produce saliva and then deliver to the oral cavity, multiple elements remain to be recapitulated in salivary gland organoid models. While *α*-amylase and AQP5 expression by acinar cells has been induced in several organoid models, some loss the expression during a quite short maturity [50]. Until recently, a model with neural cells and neuotrophic factor, neurturin input into a fetal mesenchyme containing laminin-111 extracellular matrix supporting an innervated branching epithelium was reported by Vining and colleagues [51], and it is noteworthy that abundant basal progenitors remained close proximity to nerves; moreover, the proacinar cells exhibited a prolonged maturing period mimicking that in vivo spatiotemporally. The mechanism of bidirectional interaction between nerve and epithelial progenitor cells was verified by this coculture organoid model, the highlight of researches on branching morphogenesis, and acinar cell function maintenance [23, 52].

As saliva secretion from acini depends both on membrane transport of acinar cells and actomyosin-mediated contraction of myoepithelial cells, salivary gland organoids can also be used to identify Ca2^+^-dependent mechanisms that drive myoepithelial cell contractility. A functional model was developed using a bottom-up approach, when isolated human salivary myoepithelial cells were added into adult stem/progenitor cell derived spheroids in HA hydrogel, and they self-assembled around the spheroids; more importantly, the newly formed spheroid retained responding ability when stimulated by neurotransmitters [53]. Compared to acinar and myoepithelial cells, there are relatively less information of niche factors that induce ductal cell differentiation in organoids, and thus far, no elongated network with branching morphology of ductal cells has been obtained.

### 3.3. Salivary Gland Organoids for Regenerative Medicine

Aiming to replace (or aid to regenerate) the functions of injured or diseased tissues, regenerative medicine has gathered the endeavor of engineering scientists and physicians during the last thirty years. Salivary gland organoids containing stem/progenitor cells, acini, and ductal-like structures hold promise for providing a radical solution for xerostomia, and they have shown their capability of restoring the function of irradiation-damaged glands. The first evidence was provided by Tanaka and colleagues, after orthotopically transplanted into parotid gland-defective mice, the ESC-derived salivary rudiment connected to surrounding tissues, developed into mature phenotype, and secreted saliva by gustatory stimulation [28]. Up to date, several groups have demonstrated ASC-derived organoids' efficiency in rescuing functional loss of postirradiation glands in murine models [46, 54–57]. In these models, the traditionally used ECM-like materials extracted from animal tissues are proven to be conducive to multiple cell behaviors such as adhesion, migration, assembly, and differentiation; however, the first obstacle for translation into the clinical settings is their potential tumorigenicity and immunogenicity. Several biocompatible and/or biodegradable scaffolds and matrices have been generated to solve the problem, including inregion ones such as hyaluronic acid (HA), alginate, chitosan, silk, and synthetic ones such as poly-lactic acid, poly-lactic-*co*-glycolic acid, poly-glycolic acid, and polyethylene glycol (reviewed in [58]). An ideal material needs suitable stiffness and porosity, resembling the native extracellular matrix to support cell behavior during organogenesis. Besides these scaffold-based culture models, the striking advances in microwell culture and bioprinting platform allow salivary gland organoids formed faster and more uniformly [59–62]. Hurdles ahead concern the way organoids get connected with the existing gland, including excretory ducts, blood vessels, and nerves to ensure their long-term functional maintenance.

## 4. Conclusions and Perspectives

Salivary gland organoids allow us to recapitulate exocrine epithelial cells functionally and structurally in vitro by harnessing salivary gland cells' potential. PSC-derived salivary gland organoids containing multiple salivary gland cell lineages can be a hopeful model for salivary gland development and morphogenesis studies. To engineer more faithfully recapitulating models, continued characterization of salivary gland tissue is the cornerstone. Recent advances in the single cell transcriptome revealed the molecular identity and cellular diversity of both epithelial and mesenchymal cells of adult and embryonic mouse salivary glands [63, 64]. Although difficult to collect samples, such analyses of human would be necessary for organoid engineers. As a potential strategy for regenerative medicine, ASC-derived salivary gland organoids are facing challenges that require combined approaches of stem cell biology and bioengineering. Current salivary gland organoids are lack of vascular cells; although, microvascular endothelial cells can be cocultured with salivary gland cells [65], but insufficient to form a functional network to guarantee nutrient supply as organoids expand. Microfluidic systems and biomaterials can be incorporated in future work, and organoid transplantation into an existing vascularized bed of host animals to allow the vasculature to grow into would be a promising attempt [56]. In conclusion, salivary gland organoids provide an unprecedented manner to study salivary gland development, biology, and morphogenesis. Bioengineering holds the promise to establish salivary gland organoids more physiologically relevant and more amenable to biomedical applications.

## Figures and Tables

**Figure 1:** Salivary gland organoids can be derived from distinct origins by modulating niche factors during in vitro culture. (a) Salivary gland organoids derived from ESCs by a step-wise method that recapitulates the signaling pathways during salivary gland development. ESCs are first inducted towards oral ectoderm fate by exposure to BMP4, TGF*β*-i, BMP-i, and FGF2. These oral ectoderm aggregates with the forced expression of Sox9 and Foxc1 develop into branching structures following induction of FGF7 and FGF10. (b) Salivary gland organoids can also be generated from adult stem cells isolated from biopsies. Dissociated cells can be placed in ECM with cytokines important for organogenesis, regeneration, and development including FGF, Wnt3a, R-spondin 1, and TGF*β*-i. ESCs: embryonic stem cells; BMP4: bone morphogenetic protein 4; TGF*β*-i: transforming growth factor beta inhibitor; BMP-i: bone morphogenetic protein inhibitor; FGF: fibroblast growth factor; ECM: extracellular matrix; Sox9: sex-determining region Y (SRY) box 9; Foxc1: forkhead box C1; Wnt3a: wingless-type MMTV integration site family member 3a; R-spondin1: roof plate-specific spondin 1.

**Figure 2:** Immunofluorescence images of salivary gland organoid derived from mouse PCSs (a) and mouse embryonic salivary gland E18 (b). The ductal marker K18 (green) and the acinar cell marker AQP5 (red) were shown. Scale bars, 50 *μ*m. Arrows indicate ducts (d). Arrowheads indicate an epithelial bud (e) (immunofluorescense images taken from Tanaka et al. [28]).

## Data Availability

The data used to support the findings of this study are included within the article. Previously reported histoimmunochemistry figure data were used to support this study and are available at DOI 10.1038/s41467-018-06469-7. This prior study is cited at relevant place within the text as reference [28].
